RETRACTED

# Influence of Nanosemiconductor Materials on Thermal Stability of Solar Cells

**DOI:** 10.1155/2022/6805501

**Published:** 2022-07-04

**Authors:** Aijie Ma

**Affiliations:** Hebei Chemical & Pharmaceutical College, Shijiazhuang 050026, China

## Abstract

In order to overcome the problem of long-term stability of perovskite solar cells, the author proposes a method to study the effects of nanosemiconductor materials on the thermal stability of solar cells. In this method, *n* = 3 and *n* = 1 (C_6_H_5_(CH_2_)_2_NH_3_)_2_(CH_3_NH_3_)_n-1_Pbn I_3n+1_ two-dimensional nanoperovskite films were investigated on glass substrates and indium tin oxide (ITO) substrates, respectively, on the thermal stability. Experimental results show that the glass-based nanoperovskite PMPI_3_ film was partially decomposed into PbI_2_ after being heated at 160°C. When the temperature reaches 180°C, the film is completely decomposed into PbI_2_, and the perovskite PMPI_3_ film with ITO as the substrate is completely decomposed into PbI_2_ when the heating temperature reaches 140°C. The charge transfer between the perovskite film and the substrate is the physical reason for its easier thermal decomposition on the ITO substrate. Suggestions for improving the thermal stability of perovskite solar cell devices are given from the aspects of device design and fabrication process.

## 1. Introduction

Perovskite solar cells (PSCs) have become a research hotspot in the field of efficient utilization of solar energy due to their excellent optoelectronic properties. After more than ten years of optimization of perovskite materials and improvement of cell structure, the photoelectric conversion efficiency of single-junction PSCs has increased from 3.8% in 2009 to 25.5% certified in 2020 and is expected to become the first choice for a new generation of thin-film solar cells [1]. At present, the vast majority of PSCs use the TiO_2_ mesoporous structure as the electron transport layer. However, the perovskite material has a low pore filling rate in the mesoporous structure and a large photogenerated charge transfer resistance, which is the main reason to limit the further improvement of the performance of this type of PSCs.

At present, perovskite solar cells mainly have two basic structures: mesoscopic and planar structures. Compared with the planar structure, the PSCs of the mesoscopic structure are mainly composed of five parts: transparent electrode, electron transport layer, perovskite light absorption layer, hole transport layer, and back electrode. According to the structure of the electron transport layer, the mesoscopic structure is further divided into the mesoporous structure and the nanoarray structure. Nanoparticles in the mesoporous structure can increase light scattering, improve the solar light capture efficiency of the battery, and at the same time, has a large specific surface area, which can increase the contact area between the perovskite and the electron transport layer. This in turn improves battery efficiency. Single-crystal TiO_2_ nanorod arrays (titanium dioxide nanorod arrays, TNRAs) have unobstructed electron transport channels and through-ordered pore structure, and the one-dimensional single-crystal nanorods have fewer grain boundaries and defects. At the same time, the orderly and through pores are easy to be filled with perovskite materials, which increases the contact area between TNRAs and perovskite, which can effectively make up for the lack of TiO_2_ mesoporous structure. This has attracted the attention of many researchers [2]. However, the perovskite layers deposited on TNRAs suffer from low coverage and high defect density, and the “TNRAs/perovskite” interfacial contact is problematic. As a result, the photoelectric conversion efficiency and stability of TNRAs-based PSCs are still not ideal [3]. How to optimize the contact and energy level matching between the “TNRAs/perovskite” interface, passivate the defects of perovskite films, and further improve the performance of TNRAs-based PSCs has become an urgent problem to be solved as shown in Figure 1.

RETRACTED

## 2. Literature Review

Yu et al. fabricated *α*-CsPbI_3_ QD films that were stable in air for several months and reduced the size of the crystallites to nanoscale by preparing them into quantum dots. Thus, the phase stabilization temperature of *α*-CsPbI_3_ is well controlled. The perovskite QD photovoltaic cells were fabricated, the open circuit voltage is 1.23 V, and the efficiency is 10.77%. The efficiency did not decrease after aging for 1440 h in air, demonstrating the humidity stabilization potential of CsPbI_3_ [4]. Xin et al. used graphene oxide to cross-link quantum dots to form graphene/CsPbI_3_ films, and the graphene cross-linking restricted the position of quantum dots in order to ensure that the high surface energy characteristics of quantum dots can be exerted. The graphene layer plays a blocking role against water within the device structure, and at the same time, the higher mobility ensures the transmission of excitons. When the device was placed at 60% humidity for 5 h, the efficiency decreased by only 10% of the initial level, showing good stability [5]. Hu et al. designed a gradient particle size (GGS) CsPbI_3_ bilayer. Let ADMA interact with perovskite, and a large-grained CsPbI_3_ layer was obtained at the bottom position with high charge mobility and low density of well states. This gradient particle size not only ensures higher surface energy of the upper layer material but also ensures that the lower layer material has fewer grain boundary defects. The device operates stably for 1 000 h at room temperature and a relative humidity of 20%, with an efficiency retention of 85% [6]. Selvanathan et al. developed the spontaneous interface modification (SIM) technique, which can spontaneously organize the 2D/3D perovskite top interface without the use of weakly polar solvents, resulting in a 2D/3D multidimensional perovskite top layer. The spontaneously formed ultrathin 2D perovskite not only eliminates interfacial defects but also effectively hinders moisture permeation. Finally, the CsPbIxBr3-x all-inorganic device obtained a significant efficiency improvement, the photoelectric conversion efficiency increased from 13, from 64% to 18%, and the device life is also greatly extended. The device can still retain 81% of the efficiency when stored in air for 1000 h [7]. Dong et al. found that, compared with the traditional MDMO-PPV system, P3HT has better crystallinity, and P3HT can form longer nanowhiskers under thermal annealing conditions. On the one hand, these nanowhiskers can improve the hole mobility of the photoactive layer, and on the other hand, it has a certain inhibitory effect on the migration and aggregation of PC61BM. This finding has a positive effect on the later study of using P3HT nanowhiskers to improve the thermal stability of the device [8].

RETRACTED

Therefore, in order to further study the thermal stability of nanoperovskite materials, for improving the stability of perovskite and promoting perovskite solar cells, the application in people's life is of great significance. The authors prepared (PEA)_2_(CH_3_NH_3_)_n-1_[Pb_n_ I3_n+1_]*n* = 1 and 3 films on glass and indium tin oxide (ITO) substrates, respectively, PEA = C_6_H_5_(CH_2_)_2_NH_3_. The thermal stability of PEA_2_MA_2_Pb_3_I_10_(PMPI_3_) films and PEA2PbI_4_(PEPI) films on two substrates at different temperatures were systematically studied, MA = CH_3_NH_3_.

## 3. Research Methods

In the experiment, the glass substrate and ITO substrate (15 Ω/sq) were first put into deionized water for 15 min and then placed in anhydrous alcohol for 15 min; finally, the cleaned substrate was blow-dried with high-purity nitrogen and treated with ultraviolet ozone for 30 min to enhance the wettability of the substrate surface. The dimensions of the glass substrate and the ITO substrate are both 1.5 cm × 1.5 cm. PEAI (124.5 mg), MAI (79.5 mg), and PbI2 (345.75 mg) in a molar ratio of 2 : 2:3 were dissolved in 875 mL of DMF solvent and stirred for 5 h on a heating table at 45°C to obtain nanoperovskite PMPI3 precursor solution [9]. 400 mg of PEPI was dissolved in 635 mL of DMF solvent and stirred on a heating table at 45°C for 5 h to obtain the nanoperovskite PEPI precursor solution. PbI_2_ and MAI were purchased from Xi'an Baolite Company, and DMF was purchased from Alfa Aesar Company. Two perovskite precursor solutions were spin-coated onto the treated glass and ITO substrates, respectively, the speed of the spin coater was 4000 r/s, and the time was 30 s. Then, the PMPI3 perovskite films on the glass substrate and the ITO substrate were heated at 100°C, 120°C, 140°C, 160°C, 180°C, and 200°C for 15 min on a heating stage, respectively, the PEPI perovskite films on glass substrates and ITO substrates were heated at 100°C, 120°C, 140°C, 160°C, 180°C, and 200°C for 15 min, respectively. The above experimental operations were completed in a nitrogen-filled glove box [10].

RETRACTED

After the preparation of the samples, the absorption of these annealed films was measured, and X-ray diffraction (XRD) and photoluminescence were used to characterize the decomposition degree of perovskite in the films and the decomposition products. The absorption spectra of the perovskite films were measured with an EVOLUTION220 UV-Vis spectrophotometer, the XRD patterns were measured by a Bruker AXS DimensionD8 X-ray system, and the photoluminescence spectra were measured by an optical system built in the laboratory and excited by a laser with a wavelength of 447 nm [11].

In the process of evaluating whether the perovskite lattice is stable, we usually use the tolerance factor as the criterion for judgment. The ionic radius matching in the perovskite structure should satisfy the following formula:

(1) $$\begin{array}{c} R_{A}+R_{X}=\sqrt{2}\left(R_{B}+R_{X}\right)\cdot t, \end{array}$$

where *R*_*A*_, *R*_*B*_, and *R*_*X*_ represent the ionic radii of A, B, and *X*, respectively, *t*=1 is an ideal octahedron with a common vertex connection structure.

## 4. Analysis of Results

As shown in Figures 2(a) and 2(b), nanoperovskite PMPI_3_ thin films based on ordinary glass and ITO conductive glass, respectively, were heated at 100°C, 120°C, 140°C, 160°C, 180°C, and 200°C for 15 min after the absorption spectrum. The absorption spectrum shows that PMPI_3_ film has three absorption peaks at 601 nm, 566 nm, and 515 nm, respectively. The absorption peak at 602 nm is generated by the absorption of *n* = 3 materials, the absorption peaks at 515 nm and 566 nm correspond to the exciton absorption energies of *n* = 1 and *n* = 2 materials, respectively, and at the same time, there is obvious absorption below 602 nm. This is because the PEA_2_ (MA)_n-1_ Pb_n_ I3_n+1_ nanoperovskite with larger *n* value exists in the film. It can be seen that although the molar ratio of *n* = 3 is used to configure the solution during the preparation of PMPI_3_ films, and the films prepared by spin coating are mixed films containing nanoperovskites with various *n* values [12]. From Figure 2(a), it can be found that, after annealing at 100°C, 120°C, and 140°C, the absorption spectra of the films basically overlap without obvious changes. At the same time, when the heating temperature increases to 160°C in Figure 2(a), the three absorption peaks of perovskite still exist, but the intensity becomes weaker. These phenomena indicate that the film at this temperature has partially decomposed. When the heating temperature was increased to 180°C and 200°C, the absorption peaks at 515 nm, 602 nm and 566 nm of the film disappeared, but appeared as a rapidly changing absorption band edge at 520 nm, and the color of the film changed completely to yellow [13]. It can be seen from Figure 2(b) that when the heating temperature is 100°C and 120°C, the three absorption peaks of the perovskite are clearly displayed. When the heating temperature rises to 140°C, the decomposition of the PMPI_3_ film on the ITO substrate has been completed, and the film turns yellow completely. When the heating temperature is 160–200°C, and the absorption spectrum and the color of the film on the ITO substrate are completely consistent with those at 140°C. These phenomena indicate that the ITO-based perovskite PMPI_3_ material is completely decomposed after heating at 140°C. Combined with the above experimental results, it is found that the nanoperovskite PMPI3 film with ITO as the substrate, and it is more prone to thermal decomposition than thin films on glass substrates [14].

RETRACTED

In order to understand the process and products of thermal decomposition, the XRD of each film studied in Figure 2 was measured, and the distribution of PbI_2_ and nanoperovskite PMPI_3_ in the heat-treated films was further studied. Figures 3(a) and 2(b) show the nanoperovskite PMPI_3_ with ordinary glass and ITO conductive glass as substrates at 100°C, 120°C, 140°C, 160°C, 180°C, and 200°C, respectively, on the heating stage XRD patterns after heating for 15 min. From Figure 3(a), it is found that the films have consistent and highly similar diffraction peaks when the heating temperature is 100°C, 120°C, and 140°C, and the diffraction peaks (111) and (222) are characteristic peaks of nanoperovskite PMPI_3_. At the same time, the XRD pattern only shows the characteristic peaks of the nanoperovskite PEA_2_MA_n-1_Pb_n_ I3_n+1_ with *n* = 3. Although the characteristic peaks of *n* = 1 and *n* = 2 materials are clearly reflected in the absorption spectrum. However, it does not appear in the XRD pattern, indicating that the crystal structure of the nanoperovskite film is still determined by the material of *n* = 3, and other perovskites with different *n* values exist in the film as “impurity grains.” When the temperature was increased to 160°C, the XRD pattern showed that, in addition to the diffraction peaks specific to the nanoperovskite PMPI_3_, the diffraction peak of PbI_2_ appears at 2 *θ* = 12.7°, and the intensity of the diffraction peak of perovskite becomes weaker. When the heating temperature is 180°C and 200°C, except for the diffraction peak of PbI_2_, the film has no characteristic peaks of perovskite materials [15]. It can be seen from Figure 3(b) that when the heating temperature is 100°C and 120°C, the PMPI3 film on the ITO substrate has similar nanoperovskite PMPI_3_ diffraction peaks, and the film only has the diffraction peak of PbI_2_ at 140–200°C. In summary, it is found that the nanoperovskite PMPI_3_ film on glass substrate is partially decomposed into PbI_2_ after heating at 160°C, and when the temperature reaches 180°C, the film is completely decomposed into PbI_2_, and the perovskite PMPI_3_ film on ITO substrate is completely decomposed into PbI_2_ when the heating temperature reaches 140°C.

In the absorption spectrum of Figure 2 and the XRD pattern of Figure 3, the thermal stability of the perovskite PMPI_3_ film on the ITO substrate is worse. The reason for this phenomenon may be the same as that of the three-dimensional perovskite MAPbI_3_, it is the charge transfer between the film and the substrate, regardless of whether the perovskite loses or gains electrons, resulting in the decomposition reaction.

In order to further verify the effect of charge transfer, the above experiments were repeated with *n* = 1 nanoperovskite PEPI. The exciton binding energy in PEPI films is as high as ∼230 meV, and the quality of the films prepared from solution is relatively high; substantially, no carriers are generated in the case of photoexcitation; therefore, the general film does not contain free or bound charges [16]. So, even if the substrate is ITO, there is very little chance of charge transfer between the film and the substrate. It was found that different substrates had little effect on the thermal stability of PEPI films. When the annealing temperature is 160°C, the films have very clear X-ray diffraction structures belonging to PEPI films. This also shows that the PEPI film has high crystallinity and good quality. After annealing at 180°C and 200°C, the X-ray diffraction peaks have basically presented the PbI_2_ film structure. But comparing the absorption spectra, although the spectra of the films annealed at 180°C and those annealed at 160°C are different, there are still obvious PEPI exciton absorption peaks. The film annealed at 180°C lacks the X-ray diffraction structure, indicating that the nanocrystalline structure of the film has been destroyed, but the nm-scale PEPI grains may still exist [17].

RETRACTED

In order to further understand the effect of high temperature annealing on perovskite films, the photoluminescence spectra of PEPI films on glass substrates and PEPI films on ITO substrates were further measured.  Figure 4 shows the normalized luminescence spectrum of the thin film heated at 100–200°C [18]. Although the luminescence peak of the film annealed at 180°C is slightly broadened compared to other temperatures, it is basically at the same position, which is the luminescence spectrum of PEPI, which is consistent with the absorption spectrum. It was also proved that when the PEPI film was annealed at 180°C, although the X-ray diffraction spectrum showed that the nanocrystalline structure had been destroyed, it still had the coexistence of PbI_2_ and PEPI. Under the same experimental conditions, the film annealed at 200°C did not find obvious light-emitting structure, which may be due to the fact that although the PbI_2_ film itself can also be used as a light-emitting material, the luminous efficiency at room temperature is low, and the experimental system is not sensitive enough.

For the integrity of the experiment, the photoluminescence spectra of PMPI_3_ films on glass substrates (PMPI_3_/glass) and PMPI_3_ films on ITO substrates (PMPI_3_/ITO) after different temperature treatments were measured. The material annealed at 180°C and 200°C has no obvious light-emitting structure. The luminescence peaks of PMPI_3_/glass films are all at 780 nm, and the energy is lower than the exciton peak of *n* = 3 (602 nm) because the wavelength of the laser is 447 nm, which should be affected by the nanoperovskites with different *n* values in the film. The luminescence peak position is close to the component of *n* = ∞, that is, the luminescence peak position of MAPbI_3_, indicating that there is high-efficiency energy transfer in the film until complete decomposition. However, the PMPI_3_/ITO films show very different results. First, the luminescent structures of the films at 100°C and 120°C are basically the same as those of PMPI_3_/glass, the film at 120°C has a more obvious red shift, but it is basically around 750 nm. The luminescence peaks at 140°C and 160°C occurred at 520 nm, which were obviously consistent with the luminescence peaks of PEPI. The charge transfer with the ITO substrate led to the dissociation of the PMPI_3_ (which should also include the *n* = 2 phase) film that is prone to charge generation, but part of the PEPI grains survived, which dominated the luminescence of the film after annealing at 140°C and 160°C process [19]. At higher temperatures, PEPI also eventually dissociates to PbI_2_.

RETRACTED

The charge transfer between the perovskite layer and the ITO substrate results in excess holes or electrons in the film. When excess holes appear in the perovskite film, I^−^ will form I with the excess holes, (CH_3_NH_3_Pb)^3+^ will react with I to generate CH_3_NH_2_, HI, PbI_2_, and holes, CH_3_NH_2_ and HI will volatilize as gas, and the generated holes will continue to interact with I^−^ to promote the reaction. When excess electrons appear in the perovskite, (CH_3_NH_3_Pb)^3+^ gets electrons to generate CH_3_NH_2_ and H, H and PbI^−3^ form HI, PbI_2_ and electrons, CH_3_NH_2_ and HI volatilize in the form of gas, the generated electrons will continue, and the role of (CH_3_NH_3_Pb)^3+^ promotes the reaction [20]. Therefore, when fabricating devices based on nanoperovskite materials, the influence of electrodes needs to be considered during the annealing process of the devices, or a barrier layer of suitable thickness should be inserted between the active layer and the electrodes, for example, Sb_2_S_3_, it is possible to improve the thermal stability of the device without affecting the photocurrent [21].

## 5. Conclusion

The stability of nanoperovskite PMPI_3_ thin films with ordinary glass and ITO conductive glass as substrates at different temperatures was investigated, the experimental results show that PMPI_3_ film on glass substrate is partially decomposed into PbI_2_ after heating at about 160°C for 15 min, at the heating temperature of 180°C and higher, the film is basically completely decomposed into PbI_2_, and the film on the ITO substrate begins to partially decompose into PbI_2_ in the temperature range of 120–140°C. When the temperature was raised to 140°C, the perovskite film was completely decomposed into PbI_2_. Therefore, it can be considered that the thermal stability of nanoperovskite PMPI_3_ on ordinary glass substrate is significantly better than that of perovskite on ITO substrate. For the integrity of the experiment, the thermal stability experiments of nanoperovskite PEPI films on two substrates were performed. By comparing the experimental results, it is found that the thermal stability of the nanoperovskite PMPI_3_ film based on ITO is worse than that of the film on the glass substrate, and the thermal stability of the nanoperovskite PEPI film on the two substrates is different. Combining the two experimental results, it is believed that the charge transfer between the perovskite material and the substrate may lead to the deterioration of the thermal stability of the perovskite film.

RETRACTED

## Figures and Tables

**Figure 1:** Flow chart of thermal stabilization of solar cells.

**Figure 2:** Absorption spectra of PMPI_3_ films treated at different temperatures. (a) PMPI_3_/glass. (b) PMPI_3_/ITO.

**Figure 3:** XRD patterns of PMPI3 films treated at different temperatures. (a) PMPI_3_/glass. (b) PMPI_3_/ITO.

**Figure 4:** PL spectrum.

## Data Availability

The data used to support the findings of this study are available from the corresponding author upon request.
